The article "Visual Effects of Haptic Feedback Are Large but Local" was published in 2011. Journal: PLoS One.

# Visual Effects of Haptic Feedback Are Large but Local

**DOI:** 10.1371/journal.pone.0019877

**Published:** 2011-05-10

**Authors:** Xin Meng, Qasim Zaidi

**Affiliations:** Graduate Center for Vision Research, State University of New York College of Optometry, New York, New York, United States of America; University of Regensburg, Germany

## Abstract

Vision generally provides reliable predictions for touch and motor-control, but some classes of stimuli evoke visual illusions. Using haptic feedback on virtual 3-D surfaces, we tested the function of touch in such cases. Our experiments show that in the perception of 3-D shapes from texture cues, haptic information can dominate vision in some cases, changing percepts qualitatively from convex to concave and concave to slant. The effects take time to develop, do not outlive the cessation of the feedback, are attenuated by distance, and drastically reduced by gaps in the surface. These dynamic shifts in qualitative perceived shapes could be invaluable in neural investigations that test whether haptic feedback modifies selective activation of neurons or changes the shape-tuning of neurons responsible for percepts of 3-D shapes.

## Introduction

Perceiving the correct shapes of objects is necessary for inferring object qualities, manipulating tools, avoiding obstacles, and other aspects of functioning successfully in the world. Since observers can estimate object properties from larger distances using vision than they can from touch, generally vision makes predictions that touch relies on, such as the shape of a handle or chair. However, since the information in retinal images is inherently under-determined, the inferential power of vision arises from employing intelligent heuristics/assumptions/priors, but this inevitably leads to illusory percepts in some cases. What are the possible functions of touch in such cases? Observers could rely entirely on the haptic percept and ignore the erroneous visual percept, or touch could temporarily correct the visual percept, or there could be longer lasting effects if observers learn to change their visual prior assumptions [1] and/or weights for different visual cues [2]. We tested these possibilities by measuring the effects of various types of haptic feedback on the perception of images that evoke incorrect visual percepts despite being proper perspective projections of 3-D surfaces.

Fig. 1a demonstrates that observers perceive veridical 3-D shapes when looking at perspective projections of half-cycles of a sinusoidal corrugation covered with a plaid texture [3]. However, identical shapes covered by a random-dot texture evoke qualitatively incorrect percepts (Fig. 1b), as both concave and convex surfaces are perceived as convex, while the right-slant and the left-slant are perceived as concave [4]. We have shown that both correct and incorrect percepts can be understood by first parsing the images in a manner similar to striate cortex, i.e. in terms of local orientations and spatial frequencies, and then considering flows formed from local orientations and gradients of local spatial frequencies [3], [4], [5]. The plaid textures are composed of a horizontal sinusoidal grating added to a vertical sinusoidal grating. In the images of the 3-D shapes, the horizontal component of the plaid projects to patterns of orientation flows that are distinct for the four curvatures, and the flows automatically evoke veridical shape percepts [5]. The images of the random-dot textured surfaces do not exhibit the orientation flows, but contain spatial-frequency gradients similar to the gradients of the vertical component of the plaid. Spatial-frequency gradients in an image can result from variations in surface distance or slant. In the absence of orientation flows, the perceived 3-D shapes are consistent with the prior assumption that low and high frequencies result solely from closer and more remote regions: in Figure 1b, concave and convex surfaces are seen as convex (high-low-high horizontal gradients of spatial frequency), while right and left slants are seen as concave (low-high-low gradients) [4]. In perceiving 3-D shapes, the visual system seems to ignore the distortions of the circular dots to elliptical, despite the fact that these distortions are due solely to changes in slant not distance, and could potentially disentangle the two influences on spatial frequency gradients. In other words, despite the stimuli in Fig. 1b being ecologically valid, observers do not perceive veridical shapes. We tested whether touch can “correct” the visual percepts [6] in Fig. 1b, and if observers can learn to dissociate spatial-frequency gradients from distance after repeatedly touching the surfaces.

The article "Visual Effects of Haptic Feedback Are Large but Local" was published in 2011. Journal: PLoS One.

**Figure 1:** Veridical and non-veridical percepts of 3-D shapes conveyed by surface textures. (A) Flat fronto-parallel surface and half-cycles of a 3-D vertical sinusoidal corrugation covered with horizontal-vertical plaid textures. (B) Identical surfaces covered with random-dot textures.

## Results

### Experiment 1: Haptic information can dominate vision

In normal functioning, visual percepts are often used to make predictions for tactile properties like soft, stiff, brittle, sharp, dull, sticky, or slippery, whereas touch is rarely used to make predictions for visual percepts [7]. In this experiment, we identify classes of conditions where haptic feedback can influence the visual percept, and classes where it cannot. Four half-cycles of 3-D vertical sinusoidal corrugations (Convex, Concave, Right-slant, and Left-slant) covered with random dot textures were projected in perspective (Fig. 1b). The observers viewed the 8×8° images at the proper distance through a monocular aperture, while actively “touching” the virtual 3-D surface with a SensAble PHANTOM Omni stylus (Fig. 2). A mirror was used to locate the visual image and the haptic feedback in the same plane. A red cursor on the image continuously showed the position of the stylus, enabling observers to visually locate the part of the surface they were touching. Observers were required to touch the stimuli between two red squares on the left and right edge of the center of each stimulus. The PHANTOM was set to one of three conditions: (i) No haptic feedback; (ii) haptic feedback consistent with simulated 3-D shape; (iii) haptic feedback opposite to simulated 3-D shape (concave↔convex; r-slant↔l-slant). Each trial was 100 sec. Every 10 sec there was a beep to prompt the observers to say whether they saw the shape as convex, concave, right-slant, left-slant, or flat, and either deep or shallow. Each session contained every trial condition randomly interleaved. NOTE: In the absence of a visual stimulus, when observers were instructed to touch each virtual surface between two landmarks for 40 secs, they reported veridical percepts on 97 to 100% of the trials (10 trials per shape for each of 3 observers), so we know that the haptic feedback conveys the intended shapes.

**Figure 2:** Schematic of the visuo-haptic apparatus. Through a monocular aperture, the observer viewed the sinusoidal corrugations with random-dot textures simulated on an LCD monitor, imaged by a mirror at the same location as force-feedback to the observer's finger generated by a PHANTOM stylus.

Results from 20 trials (5 observers×4 trials) per shape-feedback condition, are summarized in Fig. 3. For each response interval, the shape of the symbol represents the most frequently reported shape, and the size of the symbol represents the proportion of the 20 trials on which observers reported the majority shape (Fig. 3a). In the trials without haptic feedback (Fig. 3b), on the majority of the trials, observers perceived concavities and convexities as convex, and both slants as concave. In the trials that provided continuous haptic feedback consistent with the simulated shape (Fig. 3c), observers' visual percepts were already different from the no-feedback condition after 10 secs of touching, and as the trial progressed, they started perceiving the concave and slanted surfaces “correctly” with increasing frequency. In the trials that provided haptic feedback opposite to the simulated surface (Fig. 3d), the observers' percepts changed to the shape indicated by the haptic feedback, i.e. opposite to the previous condition. It is interesting that visual percepts develop with similar time-courses in the two haptic-feedback conditions, this can be seen by comparing similar shaped triangles in Fig. 3c and 3d across progressive response intervals.

The article "Visual Effects of Haptic Feedback Are Large but Local" was published in 2011. Journal: PLoS One.

**Figure 3:** Results of Experiment 1. (A) Symbols: Most frequently reported shape (4 trials×5 observers). Size: Proportion of majority responses per condition. Data panels show majority shape reported at each prompt after a 10 sec interval when viewing sinusoidal corrugations covered by random-dot texture without haptic feedback (B), with haptic feedback consistent with simulated 3-D shape (C), and with haptic feedback opposite to 3-D shape (D). Without haptic feedback, the observers generally perceived concavities and convexities as convex, and both slants as concave; With haptic feedback consistent with the simulated surface, observers gradually started perceiving the concave and slanted surfaces “correctly”. With the haptic feedback opposite to the simulated surface, the observers gradually perceived the surface indicated by the haptic feedback. (E) Shapes reported when viewing sinusoidal corrugations covered by random-dot texture with flat fronto-parallel haptic feedback. This feedback failed to modify the pre-training percept. (F) A flat fronto-parallel surface textured with random dots was tested with convex, concave, right-slant and left-slant haptic feedback. The curved or slanted haptic feedback did not alter the percept of the flat stimulus. (G) When the simulated surfaces were covered by a plaid texture, the observers could perceive the shape correctly, and haptic feedback opposite to the shape did not alter the visual percept.

Notice that when haptic information changed the visual percept, it did not over-ride the texture cue. The final percepts in Fig. 3c corresponded to the simulated surfaces, so the texture cues were physically compatible with the final percepts. In addition, in the absence of orientation cues, the spatial frequency gradients depend on the magnitudes of the slants, but not their directions, so the images of the concave and convex surfaces are very similar, as are the images of the two slants, therefore the final percepts in Fig. 3d also do not over-ride texture cues. To test whether haptic feedback could create visual percepts at odds with visual cues, we used three additional conditions: (i) flat fronto-parallel haptic feedback was combined with the images of the random-dot curved and slanted surfaces, (ii) a random-dot flat fronto-parallel surface was coupled with convex, concave, right-slant, and left-slant haptic feedback, (iii) Convex, Concave, Right-slant, and Left-slant corrugations covered by plaid textures, which observers perceive as correct 3-D shapes, were presented with haptic feedback opposite to each simulated shape. The summary figures, show that in all of these conditions the feedback failed to modify the initial visual percept prior to haptic feedback. The shape reports under flat haptic feedback (Fig. 3e) were essentially the same as under no haptic feedback, and the curved haptic feedback did not change the flat percept of the images simulating flat surfaces (Fig. 3f). Finally, the “opposite” haptic feedback did not change the percepts of the images with plaid textures that contain orientation cues to the veridical shapes (Fig. 3g).

The article "Visual Effects of Haptic Feedback Are Large but Local" was published in 2011. Journal: PLoS One.

Could the effects of haptic feedback be understood in terms of statistically optimal cue combination [8]? In the absence of haptic feedback, Fig. 3a shows that observers perceive the random-dot concave surface predominantly as convex, but only on about 54% of the trials, and the two slants as concave on about 73% of the trials, whereas in the absence of visual stimulation, haptic feedback evoked the intended percept on 97–100% of the trials. A Bayesian observer would give greater weight to the lower variance (more reliable) percepts [9], so in the case of conflict between visual and haptic percepts would be more likely to modify the less reliable visual percept. In the case of the flat feedback with the curved visual surfaces (Fig. 3f), these surfaces were never reported as flat without feedback, so the feedback did not modify the visual percept from 3-D to flat. Similarly, since there was almost no variance in the initial visual percepts prior to haptic feedback of the flat surfaces (Fig. 3g) and the non-concave surfaces with plaid textures (Fig. 3h), haptic feedback had little effect.

All of the shape-feedback conditions in Experiment 1 were randomly mixed in each session, so we presume that observers were using the same criteria to report what they saw in all the trials. The results show that haptic feedback reliably altered the visual percept in some of the conditions (Fig. 3c,d), but in others the reported shapes were different from those simulated by haptic feedback (Fig. 3e–g), confirming that observers' reports reflected not the shape that they touched, but rather the shape they saw as per the instructions.

### Experiment 2: Temporal limits of visual effects of haptic feedback

While running Exp 1, we noticed that even after 100 sec of continuous touching, as soon as we stopped touching the virtual surface, the effect of the feedback vanished. To quantify this effect, we used the L-slant and R-slant stimuli with random-dot textures (The two right-most panels in Fig. 1b). Observers were asked to first report the perceived shape after looking at it for 5 secs. They then touched the virtual surface for 40 secs with veridical haptic feedback (consistent with the simulated 3-D shapes but inconsistent with the initial percepts of concavity), and reported the perceived shape 0, 5, 10, and 15 secs after cessation of feedback (i.e. 45, 50, 55 & 60 secs after the beginning of each trial). There were 5 trials per condition for 3 observers. The combined results plotted in Fig. 4, show that before haptic feedback, both slanted surfaces were perceived as concave. After 40 secs of veridical haptic feedback, each slant was perceived correctly on over 90% of the trials, but 5 secs after cessation of feedback, the percept started to change, and after 15 secs the reported shape had reverted to the pre-feedback percept. We had hoped that visual system would use the haptic feedback to learn that the frequency gradients in the images actually signaled slant rather than distance, and would learn to correlate the elliptical shapes of the texture elements with the surface angle indicated by touch, so the temporary nature of the effect was disappointing, and suggested an absence of perceptual learning or other lasting neural modification.

The article "Visual Effects of Haptic Feedback Are Large but Local" was published in 2011. Journal: PLoS One.

**Figure 4:** Results of Experiment 2. (A) Symbols: Most frequently reported shape (5 trials×3 observers). Size: Proportion of majority responses per condition. (B) Data panel shows majority shape reported when viewing L-slant and R-slant sinusoidal corrugations covered by random-dot texture with haptic feedback consistent with simulated 3-D shape. Observers viewed the stimulus for 5 sec without haptic-feedback, reported the shape, then touched the stimulus for 40 sec, reported the shape, and then made reports every 5 secs without any additional haptic feedback.

### Experiment 3: Spatial limits of visual effects of haptic feedback

Given that the visual effects of haptic feedback were temporary, we then tested whether the effects of haptic feedback could propagate over space, and across interruptions in the simulated surface. Left-slant and Right-slant surfaces covered by random dots from Fig. 1b were modified to the stimuli in Fig. 5a to test any possible attenuation of feedback effects due to distance between locations of touching and seeing, versus the effect of interrupting the surface by a gap. Observers were provided haptic feedback consistent with the simulated 3-D shapes, i.e. inconsistent with the initial percepts of concavity, and asked to report the shape between the two green dots while moving the Phantom cursor between the two red dots, thus keeping a constant distance of 3.98 deg between locations of touching and seeing, with or without a gap of 0.53 deg. On each trial, the observer reported the shape after touching the surface for 40 secs. Fig. 5c summarizes the results for 3 observers times 10 trials for each condition. It is clear that if touch and vision are on a continuous surface, the effect of the feedback, i.e. a switch from a concave to slanted percept, propagates over 3.98 deg, but is considerably reduced compared to when people were looking where they were touching (from over 90% veridical after 40 sec of touching in Fig. 3c to 57% veridical in Fig. 5c after the same feedback interval by the same observers). If a gap interrupts the surface between the touch and vision locations, the effect of the feedback is drastically reduced: the reported percept of the R-slant remained concave, while the reported percept of the L-slant varied between flat and concave.

The article "Visual Effects of Haptic Feedback Are Large but Local" was published in 2011. Journal: PLoS One.

**Figure 5:** Results of Experiment 3. (A) Experiment 3 stimuli: Left-Slant and Right-Slant surfaces covered by random dots, with or without a gap of 0.53 deg in the center. The red squares indicate the location of touching, and the green squares the location of looking. (B) Symbols: Most frequently reported shape (10 trials×3 observers). Size: Proportion of majority responses per condition. (C) Data panel shows shape reported most frequently when viewing L-slant and R-slant sinusoidal corrugations covered by random-dot texture after 40 sec of haptic feedback consistent with simulated 3-D shape. The effect of haptic feedback propagates over the continuous surface although reduced considerably, but is attenuated drastically when a gap interrupts the surface.

## Discussion

This study follows from earlier results showing statistically significant effects of haptic feedback on the weighting of texture versus disparity cues [2], and on the “light from above” prior assumption [1], in perception of 3-D shape from static images. The light prior study showed that proportion of observers' percepts reported as convex or concave spheres, changed as their assumptions about light position were altered by haptic feedback. Our results are compatible with observers giving greater weight to the haptic information where it was more reliable than the visual information, but the temporary nature of the perceptual modification (Fig. 4) makes it unlikely that observers changed their prior assumption that spatial frequency is a cue to distance not slant, or learned to increase the weight of the change in element shape from circular to elliptical as a cue to slant. The lack of a substantial lasting effect in our experiments, may also explain why the effects of haptic learning on the weighting of different visual cues were extremely small when measured after cessation of feedback [2], i.e. showing a statistically significant difference in slopes, but overlapping error bars for all the individual comparisons.

The article "Visual Effects of Haptic Feedback Are Large but Local" was published in 2011. Journal: PLoS One.

The visual effects of haptic feedback in this study were local in time and space. Similarly, a flat curved object that appears curled in monocular viewing (Fig. 6), appears to become flat around the part of the front edge that is being touched, but reverts to curled when not being touched [10]. Since vision functions over longer distances than touch, during everyday activities, vision generally provides predictions for touching, grasping, stepping, sitting down etc. Consequently, vision is sometimes claimed to dominate touch [11], but our experiments show that haptic feedback can substantially alter visual percepts when the visual percepts are less reliable than the haptic percepts. On the other hand, our demonstrations of the temporary nature of haptic dominance, and the lack of substantial visual learning from haptic feedback, argue against Berkeley's notion of the primacy of touch for spatial awareness [6]. Instead, it seems that the nervous system dynamically weighs the reliability of disparate signals in reaching a percept.

**Figure 6:** Visuo-haptic interactions with a real object. Griffiths & Zaidi [7] showed that a real flat object with curved edges appears curled in monocular viewing, but the percept can be corrected locally while touching the front edge. To view the illusion, with one eye covered, the shape (A) is held directly in front of the observer, with the straight edges parallel to the line of sight. The shape is then slowly raised until the line of sight is elevated from the horizontal by approximately 45°. The physically flat object then appears to be curled upwards. If the observer holds the object at the tips of the curved edge with both hands, the strength of the illusory percept is reduced, showing that haptic depth information interacts with visual cues. In addition, it is possible to break the illusion by running a finger along the closest edge of the object. If an observer touches one end of the closer curved edge, it is still possible to see the opposite end of the stimulus as having an illusory curl. If the observer then slowly runs a finger along the closer curved edge, the illusion gradually disappears around the region closest to the finger, but returns in the wake of the finger's passage. The effect of the haptic feedback in diminishing the illusory percept is thus local and temporary.

The article "Visual Effects of Haptic Feedback Are Large but Local" was published in 2011. Journal: PLoS One.

An increasing number of intriguing interactions between touch and vision have been documented recently [12], [13], [14]. Parallel to our work are demonstrations of perceiving two flashes from a single flash presented concurrently with two brief tactile stimuli [15], resolving the perceived rotation of a motion defined sphere by touching a real rotating sphere [16] and resolving binocular rivalry between oriented Gabors by touching a real grooved stimulus [17]. The importance of co-ordination between visual and haptic percepts has generated a search for neural substrates at the single-cell [18], [19] and cortical area levels [20], [21], [22]. Shape analysis is a necessary pre-semantic component of object recognition. The robust and specific changes in qualitative 3-D shapes shown in this study could be especially useful in neural investigations. In particular, it would be interesting to decipher whether the dynamic shifts from perceived convexity to concavity are due just to shifts in activation of individual neurons in population coding analyses, or whether they involve changes in shape-tuning of neurons selective for 3-D object shapes [23].

## Materials and Methods

### Apparatus and stimuli

The stimulus was shown on a 23′ wide screen flat panel LCD monitor. The vertical refresh rate was 60 Hz, and the spatial resolution was 2048 by 1152 pixels. In a dark room, the observers viewed the stimulus in a mirror through a monocular aperture from a distance of 53 cm. The haptic stimulus was created by a force-feedback PHANTOM Omni stylus. The stylus was attached to the index finger of the observer's dominant hand, such that the tip of the stylus coincided in position with the tip of the finger. The stylus thus followed the movements of the finger. An appropriate force was applied to the tip of the stylus when it reached the position of the simulated haptic surfaces, creating a compelling sensation of touching a solid surface with the finger. To view the stimulus, the observer's line of sight was pitched 70° downward. The LCD monitor was slanted 20° up from horizontal. So the line of sight was perpendicular to the image plane (Fig. 2). A chin and forehead rest limited head movements.

In Exp 1, each of four half-cycles of 3-D sinusoidal corrugations (Convex, Concave, Right-slant, and Left-slant), covered with plaid or random dot textures, were projected in perspective (Fig. 1a, b). Observers viewed the stimuli as 8×8° images. A red cursor on the image showed the current position of the stylus. Observers were instructed to touch the surface between the red squares (0.16×0.16°) on the left and right edge in the middle of each stimulus. Observers were instructed to look at the cursor when touching the surface. Exp 2 and 3 used just the Right-slant, and Left-slant half-cycles covered with random dot textures, and in Exp 3, observers were instructed to look between two green squares that were at a different location than the red squares.

The article "Visual Effects of Haptic Feedback Are Large but Local" was published in 2011. Journal: PLoS One.

### Procedures

In Exp 1, Each trial was 100 sec. Every 10 sec there was a beep to prompt the observers to report the perceived shape of the surface orally as convex, concave, right-slant, left-slant or flat, and deep or shallow. Each session contained every trial condition randomly interleaved. Observers were encouraged to take breaks between trials, each session was divided into two blocks, with a break of at least 2 mins between blocks, and unlimited rest allowed between sessions. Each observer ran 4 trials for every shape-feedback condition. The observer's task in Exp 2 and 3 was they same as in Exp 1. In Exp 2 and 3 the haptic feedback was provided for 40 secs on each trial. The details of the time-course of the shape reports and the numbers of trials are described in the main text.

### Observers

The observers in this study included both authors and four individuals who were un-informed about the purposes of the study until after data collection. All had normal or corrected-to-normal acuity. All experiments were undertaken with the understanding and written consent of each observer, and approval from the SUNY Optometry Institutional Review Board.
